# Eco-Efficiency Measurement of Green Buildings and Its Spatial and Temporal Differences Based on a Three-Stage Superefficient SBM-DEA Model

**DOI:** 10.1155/2022/3147953

**Published:** 2022-07-11

**Authors:** Wei Liu, Zhihao Ou, Cheng Lin, Zeyi Qiu

**Affiliations:** School of Civil Engineering and Architecture, East China Jiaotong University, Nanchang 330013, China

## Abstract

To explore the development of green building eco-efficiency in China, a three-stage superefficient SBM-DEA model was used to measure the green building eco-efficiency in China based on interprovincial panel data from 2013–2020, and the interprovincial and regional development patterns and evolutionary characteristics of green building eco-efficiency were analyzed from the time series and spatial dimensions. It is found that the overall level of green building efficiency in China is low, and there are significant provincial and regional differences, and the overall pattern of gradient development from medium-medium-low efficiency area to medium-medium efficiency area gradually transitions and shows significant spatial agglomeration and path dependence; among them, the spatial spillover and diffusion effect of high-efficiency areas is significant, while low-efficiency areas generally maintain low growth, and most areas have “Matthew effect,” showing the spatial club convergence characteristics that developed regions tend to be H-H agglomerative, and less developed regions tend to be L-L agglomerative. For this reason, the local governance of green buildings should be strengthened, and a cross-regional linkage development mechanism should be established to deepen the technical cooperation and division of labor between regions.

## 1. Introduction

The pace of China's new urbanization and modernization has been accelerating, and the resulting resource, environmental, and social problems have been increasing. Among them, building energy consumption and pollution seriously endanger the ecological environment and restrict the development of the industry [1]. The World Energy Organization (IEA) predicts that China's building energy consumption will reach 15.2 tce in 2030, and its energy consumption and related emissions will increase about 1∼3 times in 2050 [2]. Ecological protection plays a very important role in urbanization [3]. Obviously, the large-scale construction and urban expansion in China have gradually intensified the contradiction between economic development, energy demand, and ecological environment, and the public demand for and willingness to accept green building supply is increasing, and green building will become one of the themes of sustainable urban development in the future. With the increasing demand for urban eco-environmental protection and resource intensification, the development of green buildings in China at this stage is indeed slightly effective, and the scientific measurement of its eco-efficiency is of profound significance for the sustainable development of China's construction industry.

The concept of Eco-Efficiency is derived from a report submitted by the World Business Council for Sustainable Development (WBCSD) in 1992, and its core aims to portray the ability of a certain field (industry, region, or economy) to obtain more high-quality outputs with less resource input and effectively reduce negative environmental impacts, aiming to achieve win-win or multiwin goals [4]. In the case of green buildings, their eco-efficiency emphasizes the acquisition of higher economic or environmental value with smaller construction resources and environmental costs. Therefore, most of the existing studies on eco-efficiency in construction have focused on the economic, environmental benefits, and energy recovery aspects of green buildings, and few studies have been conducted on green building eco-efficiency itself. Chel and Kaushik [5] described the economic and environmental impacts of actual buildings before and after construction, emphasizing the importance of zero-energy building design before construction, low-energy green materials during construction, and the use of low-energy energy-efficient equipment in later stages. Chen et al. [6] used structural decomposition analysis to compare the differences in building energy consumption between the United States and China and to provide systematic ecological decision making for green buildings in China based on dimensions such as energy intensity effects and ecological effects in the building industry. Rodriguez et al. [7] assessed the eco-efficiency of Spanish buildings from the perspective of solid waste, with special emphasis on its role in further recycling of green building waste. At the level of spatial differences in eco-efficiency, domestic and international studies have mostly focused on the perspectives of urban development and regional environment. He and Hu [8] measured the eco-efficiency of an urban agglomeration (Chengdu-Chongqing) using super-Slack based on energy and environmental issues, revealing that large cities are more eco-efficient, and vice versa for small cities. From the perspective of industrial land, Deng and Tang [9] measured its eco-efficiency using super-SBM and investigated its spatial differentiation characteristics through spatial autocorrelation. Based on the DEA-Malmquist model, Chen [10] measured the industrial eco-efficiency of 31 provinces in China and measured its convergence. The empirical results show that industrial eco-efficiency has not been effective in China since 2008 and that changes in pure technical efficiency have been the main driver of industrial efficiency. The results show that industrial eco-efficiency has not been effective in China since 2008 and that purely technical efficiency changes are the main driver of industrial efficiency. Lu et al. [11] study the ecological value of green buildings from a systemic perspective, integrating a systemic game analysis framework with government, developers, and consumers as participants. By constructing a regional eco-efficiency evaluation model and using exploratory spatial statistical analysis, Qu [12] empirically measured and analyzed the spatial and temporal correlation and agglomeration characteristics of regional eco-efficiency in China and studied the driving factors of eco-efficiency changes. Liu and Yu [13] used structural equation modelling and AMOS software to construct a structural model of green building development based on survey questionnaires to explore the key influencing paths and key influencing factors driving the development of green buildings, so as to reveal the driving mechanism of green building development and propose corresponding driving countermeasures. J. R. Xu [14] examined the impact of government environmental audits on eco-efficiency using multiple regression and PSM methods. Our analysis shows that government environmental audits can significantly improve both static and dynamic eco-efficiency. Jiang and Tan [15] calculated the eco-efficiency of each region based on the econometric model of Window slacks and formed a spatial network of regional eco-efficiency spillovers from the causality model.

The widespread rise of green building helps improve the concept of urban and rural construction, reduce the constraints of building resources, and help the energy-saving and environmental protection strategy, which is of great significance and is an important vehicle to prompt the industry to move from the simple pursuit of economic benefits to the direction of improving resource utilization and ecological benefits. In recent years, the awareness of and demand for the concept of green building have gradually increased throughout society, the initial benefits of green building marketisation have emerged, the scale of layout has continued to grow, and a number of demonstration and benchmark projects have been set up, which have become an important symbol of building energy efficiency and emission reduction. Green building eco-efficiency is a judgement of the impact of green building economic activities on the ecological environment, while China's green building started late, and development is still relatively lagging behind, and there is a lack of scientific quantitative research on this. Therefore, this paper scientifically constructs an evaluation index system based on nonexpected output and reasonably measures its eco-efficiency level, providing a new research perspective and technical method for the research system to establish the measurement and analysis of green building eco-efficiency; at the same time, based on the theoretical logical perspective of national, regional, and interprovincial differences, it analyzes the spatial and temporal differences and evolutionary characteristics of green building eco-efficiency and identifies the key influencing factors driving green building eco-efficiency. It also identifies the key influencing factors that drive green building eco-efficiency, reveals the relationships among them, and explores more accurate and effective paths to improve green building eco-efficiency, with a view to providing theoretical support and practical reference for improving the decision-making mechanism of local governments, as well as providing a forward-looking strategic vision for the market's spontaneous focus on green building development, and broadening the road to sustainable and healthy development of green buildings.

## 2. Literature Review

### 2.1. Current Status of Eco-Efficiency Research

For decades, As the Chinese government attaches increasing importance to environmental protection, it has become increasingly urgent to conduct a comprehensive, quantitative, and objective assessment of eco-efficiency for sustainable development. As a result, the concept of eco-efficiency has been the subject of intense research in academic circles, and the idea of eco-efficiency has rapidly spread to many areas of society. At present, the main methods of measuring eco-efficiency at home and abroad are the single ratio method, the indicator system method, and the model method.

Although the single ratio method fits well with the eco-efficiency theory, it requires a single indicator factor, is highly subjective when converting indicators, and has poor environmental applicability, cannot correctly distinguish efficiency differences, and does not guarantee the accuracy and precision of the measurement.

The indicator system evaluation method measures the magnitude of eco-efficiency by screening the various input factors that affect eco-efficiency and establishing a system of evaluation indicators. In 2017, Özokcu and Özdemir [16] explored the relationship between environmental degradation and economic development using two empirical models through the context of the environmental Kuznets curve (EKC), and based on this, they established a system of eco-efficiency evaluation indicators. Zhang and Ye [17] focused on the concept of eco-development and innovation efficiency and integrated the PPC model in RAGA to evaluate the eco-innovation efficiency of different industrial sectors. Their findings demonstrate that the level of efficiency is limited by the intensive type of industry and clarify the important factors affecting the efficiency improvement, so as to provide a reference for the innovation development of various industries. Fu et al. [18] applied eye-tracking techniques and questionnaires within the framework of the stimulus-organism response model (SOR) and technology acceptance model (TAM) to investigate the factors influencing public acceptance of 5G base stations. Jiang et al. [19] reassessed the sustainability efficiency of Chinese listed companies based on a green perspective indicator system; concluding that there is still much room for improving the green sustainability efficiency of listed companies. Wang et al. [20] constructed a comprehensive eco-efficiency index for Jiangsu and evaluated the eco-efficiency of 13 cities through the entropy-weighted TOPSIS method. The study showed that the ecological efficiency of Jiangsu varied widely, with the highest ecological efficiency in central Jiangsu and relatively low in the north and south of the country.

The main advantage of the DEA method and its extensions is that it is scale-independent and objective; it evaluates the relative effectiveness of decision-making units (DMUs) by means of linear programming models, and it is particularly advantageous for evaluating the efficiency of participating projects with multiple inputs and outputs. The method is popular among domestic and international scholars, especially the application of DEA extension models to eco-efficiency. Yasmeen et al. [21] assessed the eco-efficiency of 30 regions in China using a superefficient DEA model and a systematic GMM approach and explored the effects of urbanization, technological innovation, and environmental regulations on eco-efficiency, showing that the eastern region ranked highest in terms of eco-efficiency. Mardani et al. [22] showed the superiority of DEA models in the field of energy efficiency when the production function between inputs and outputs is almost nonexistent or extremely difficult to obtain. Liu and Zhang [23] used an EBM-ML model with nondesired outputs to measure eco-efficiency and decomposition efficiency in 30 provinces in China from 2009 to 2018, using in-depth analysis in time and space. Zhu and Liu [24] used the superefficiency SBM-DEA model to measure eco-efficiency in Zhejiang Province and constructed a multiple linear regression model based on this model to evaluate the factors affecting eco-efficiency. The results of the multiple regression analysis showed that the positive impact of income, structural, and institutional factors on eco-efficiency was gradually weakening. Mao et al. [25] used descriptive analysis and one-way ANOVA to understand the sensitivity levels of metro passengers and to analyze their adaptive behavior based on their sensitivity to subenvironmental health risks. Chen [26] integrated the SBM-Undesirable model with the ML index to measure and analyze the level of green energy efficiency, to clarify the different relationships between the role of technological advances on regional energy efficiency, and to reveal the spatial spillover effects of different external environmental variables. Zou et al. [27] considered the division of nonenergy and energy inputs based on the use of nonuniform proportional reduction in order to construct and assess the production possibility set of energy efficiency environmental efficiency of Chinese provinces and cities, and they used an improved DEA model to calculate the efficiency level of Chinese provinces and cities in 2016. Zhan et al. [28] used the Malmquist-DEA index to evaluate and explore the differences in eco-efficiency of marine rangelands in different regions. Chen [29] integrated meta-frontier data envelopment analysis (DEA) and inclusive eco-efficiency and proposed a modified meta-frontier relaxation-based metric model (SBM) model and a meta-frontier nonradial directional distance function (NRDDF) model.

### 2.2. Current Status of Research on Spatial and Temporal Differences

At present, foreign studies on spatial and temporal differences in eco-efficiency are mainly focused on two levels: the analysis of the characteristics of differences and the causes of differences. Based on the perspective of urban agglomeration development, Chang et al. and Ren et al. [30, 31] measured urban eco-efficiency in the process of urbanization development and studied the spatial and temporal differences in urbanization eco-efficiency between regions and its influencing factors. Zhang et al. and Han et al. [32, 33] explored the spatial and temporal differences and evolutionary characteristics of industrial eco-efficiency in regional urban agglomerations, emphasized the spatial spillover effects of neighboring cities, and put forward reasonable suggestions for ecological green development based on the research results. Ho et al. [34] analyzed the spatial distribution and convergence characteristics of the eco-efficiency of Chinese provinces and cities. Yu et al. [35] conducted an empirical examination of the eco-efficiency of key environmental protection prefecture-level cities in China from 2003 to 2015 to analyze the spatial and temporal differences in eco-efficiency of cities in different regions and provide insights for decision makers to quantitatively assess the sustainable development of cities. To explore the growth paths of green cities in China, Huang and Hua [36] used two improved DEA methods and spatial modelling to examine the convergence patterns of ecological efficiency in different heterogeneous cities, aiming to achieve an effective balance between economic growth and environmental protection in green cities. The causes of differences mainly refer to the influencing factors that cause spatial and temporal differences. Overseas studies on the influencing factors of spatial and temporal differences in eco-efficiency have mostly focused on policy, materials, and technology. At the policy level, Ragheb et al. [37] analyze the impact of the introduction and practice of “green building systems” on local eco-efficiency differences based on local policy differences. In terms of green building materials and technologies, Sposito and Scalisi [38] highlight the important contribution of sustainable building materials and green technologies to the difference in eco-efficiency set in the construction industry. Thomassen et al. [39] introduce a green technology indicator evaluation system to assess the technical, economic, and environmental potential of emerging green technologies in different geographical areas at different stages of technological development in order to achieve minimum environmental impact and maximum economic impact.

Domestic studies on the factors influencing spatial and temporal variation in eco-efficiency have mainly focused on the macro level and the perspectives of urban construction, technological progress, and multiparty games. In terms of macro-level changes in eco-efficiency, Wu et al. [40] measured and analyzed industrial eco-efficiency in 31 provinces in China using provincial-level panel data and then explored the factors affecting efficiency; the results showed that industrial eco-efficiency in three provinces and cities showed a steady upward trend in the time series, but there were significant differences in regional cross-sections. Li et al. [41] used the SBM model to measure the eco-efficiency of four special economic zones, 78 general cities, and 13 metropolitan cities, which were analyzed using the SBM model to analyze the spatiotemporal evolutionary characteristics, as well as the differences across regions; the study showed that the eco-efficiency of most cities was highly variable, and the degree of urban coordination was low. Tang and Meng [42] used panel data to measure eco-efficiency in 26 provinces and cities and analyzed its evolution and heterogeneity pattern based on regionalization; the results showed that eco-efficiency in China has significant spatial correlation and interprovincial clustering characteristics. Based on the spatial and temporal differences and variability of regional and interprovincial eco-efficiency, Ren et al. [43] constructed a spatial econometric model to examine the key drivers of eco-efficiency and its evolution and clarified the mode of action and degree of influence of internal and external drivers. At the urban construction level, Song et al. [44] used the double difference method (DID) to evaluate the impact of low-carbon city construction on urban eco-efficiency and explored the differential impact based on heterogeneous resource dependence and city size. Lu and Fang [45] measured the eco-efficiency of urban construction land and quantitatively analyzed the spatial pattern and the impact characteristics of its elements. Man et al. [46] quantified environmental regulation policies and explored the impact of environmental regulation on regional eco-efficiency using four urban agglomerations in eastern China as research objects. Li and Wang [47] argue that technological progress can be achieved by increasing the level of technology and acting on total factor productivity and demonstrate that regional differences in eco-efficiency in China's construction industry are caused by the degree of technological progress. At the level of multiplayer games, Wang [48] analyzes the tendency of two influential players to choose green buildings to enter the market under the premise of government subsidies, based on evolutionary game theory.

Through careful combing of research results at home and abroad, it can be seen that, as an important carrier of sustainable urban development, the eco-efficiency of green buildings is the best balance between the pursuit of resource demand, economic benefits, and ecological values in the construction industry, but in the existing research on eco-efficiency, it is more applied to industry, agriculture, etc. The research and application results on the eco-efficiency of green buildings are also relatively weak, and there is even a lack of research and application results based on green buildings themselves. There is a lack of systematic analysis based on green buildings themselves and the regional economic context they are based on. Therefore, this study focuses on the input-output situation of building value output and environmental load, combines the three-stage DEA model and superefficient SBM model to measure green building eco-efficiency, and uses kernel density estimation, Moran's I index, and its scatter plot to analyze the regional differences, agglomeration characteristics, and spatial and temporal evolution patterns of green building eco-efficiency.

## 3. Research Methodology and Theoretical Model

### 3.1. Three-Stage Superefficient SBM Model

Considering the special characteristics of green building eco-efficiency measurement such as variable market environment, inaccurate value information, and large random errors, the traditional DEA method has been difficult to meet the measurement requirements. In this paper, the superefficient SBM model is used to improve the three-stage DEA model for efficiency measurement, which solves the defect of not being able to further evaluate the efficiency level of an effective decision-making unit (DMU) and can effectively eliminate the influence of environmental variables and random factors, so as to obtain more realistic and accurate measurement results. The model is constructed in the following three steps.

#### 3.1.1. Stage 1

Construct the superefficient SBM model. Draw on the superefficient SBM model improved by Tone [49] on the basis of the nonexpected output SBM model, the DMUs on the production frontier of the same data envelope can be effectively distinguished, and the initial efficiency value and input slack value of each DMU are measured based on the input-output data. The model is as follows:

(1) $$\begin{array}{c} \rho =\min\frac{1/m\sum_{i=1}^{m}{\bar{x}}_{i}/x_{i0}}{1/\left(s_{1}+s_{2}\right)\left(\sum_{r=1}^{s_{1}}{\bar{y}}_{r}^{a}/y_{r0}^{a}+\sum_{j=1}^{s_{2}}{\bar{y}}_{j}^{b}/y_{j0}^{b}\right)},\\ \text{s.t.}\left\{\begin{array}{c} x_{0}=X\lambda +S^{-},\\ y_{0}^{a}=Y^{a}\lambda -S^{a},\\ y_{0}^{b}=Y^{b}\lambda -S^{b},\\ \bar{x}\geq \sum_{j=1,\neq 0}^{n}\lambda_{j}x_{j},\\ {\bar{y}}^{a}\leq \sum_{j=1,\neq 0}^{n}\lambda_{j}y_{j}^{a},\\ {\bar{y}}^{b}\leq \sum_{j=1,\neq 0}^{n}\lambda_{j}y_{j}^{b},\\ \bar{x}\geq x_{0},\\ {\bar{y}}^{a}\leq y_{0}^{a},\\ {\bar{y}}^{b}\geq y_{0}^{b},\\ \sum_{j=1,\neq 0}^{n}\lambda_{j}=1,\\ S^{-}\geq 0,\\ S^{a}\geq 0,\\ S^{b}\geq 0,\\ {\bar{y}}^{g}\geq 0,\\ \lambda \geq 0, \end{array}\right. \end{array}$$

where *n*, *x*, *m* are the number of decision units, input items, and input indicators, respectively; *y*^*a*^, *y*^*b*^ are the expected output items and nonexpected output items, respectively; *s*_1_, *s*_2_ are the number of indicators of the first two, respectively; *s*^−^, *s*^*a*^ and *s*^*b*^ are the slack variables for inputs, expected outputs and, nonexpected outputs, respectively; *λ* is the weight vectors, and *ρ* are the objective function values, that is, the eco-efficiency values of green buildings, with *ρ* ≥ 1 indicating that the DMU is valid and *ρ* < 1 indicating that the DMU is invalid, and improvements need to be made to the inputs and outputs.

#### 3.1.2. Stage 2

Construct the stochastic frontier model (SFA). Draw on the SFA regression model proposed by Fried et al. [50], and the cost function model for decomposing the input slack values obtained in stage one, so as to remove the disturbances caused by the external environment, random errors, and other factors as follows.

(2) $$\begin{array}{c} S_{ni}=f\left(Z_{i};\beta^{n}\right)+\nu_{ni}+\mu_{ni};\;i=1,2,\ldots ,I;\;n=1,2,\ldots ,N, \end{array}$$

where *s*_*ni*_ is the input slack value of the first *n* term of the first DMU; *Z*_*i*_=(*Z*_1*i*_, *Z*_2*i*_,…*Z*_*pi*_) is the P environmental variables, *β*^*n*^ is the parameter to be estimated for *Z*_*i*_, and *f*(*Z*_*i*_; *β*^*n*^) is the effect of the external environment on the input slack value; *ν*_*ni*_+*μ*_*ni*_ is the mixed error term, *ν*_*ni*_ is the random error term, and *ν* ~ *N*(0, *σ*_*v*_^2^) is assumed; *μ*_*ni*_ is the management inefficiency term, and *μ* ~ *N*^+^(0, *σ*_*μ*_^2^) is assumed, and *ν*_*ni*_ and *μ*_*ni*_ are independently uncorrelated. To achieve the removal of the effects of the external environment and random errors, the inputs are adjusted as follows:

(3) $$\begin{array}{c} X_{ni}^{A}=X_{ni}+\left[\max\left(f\left(Z_{i};{\hat{\beta }}^{n}\right)\right)-f\left(Z_{i};{\hat{\beta }}^{n}\right)\right]+\left[\max\left(\nu_{ni}\right)-\nu_{ni}\right], \end{array}$$

*X*_*ni*_^*A*^ is the adjusted input value, and *X*_*ni*_ is the input value before adjustment, $\left[\max\left(f\left(Z_{i};\hat{\beta^{n}}\right)\right)-f\left(Z_{i};\hat{\beta^{n}}\right)\right]$ is the external environment adjusted to the same state, and [max(*ν*_*ni*_) − *ν*_*ni*_] is the random error adjusted to the same state.

#### 3.1.3. Stage 3

Based on the adjusted input and original output data, the superefficiency SBM model is then used to measure the efficiency value, which is relatively true to reflect the actual management level of the DMU.

### 3.2. Kernel Density Estimation Method

Kernel-Density estimation is a nonparametric evaluation method used to estimate the probability density of a random variable by calculating a continuous kernel density curve to depict the distribution extension of the random variable [51]. The expression of its density function is given by the following equation:

(4) $$\begin{array}{c} ①\;f\left(x\right)=\frac{1}{Nh}\sum_{i=1}^{N}K\left(\frac{X_{i}-\bar{x}}{h}\right),\\ ②\;K\left(x\right)=\frac{1}{\sqrt{2\pi }}e^{-\left(x^{2}/2\right)}, \end{array}$$

where *N* is the number of samples, *h* is the bandwidth, which is used to control the smoothness of the density curve; Xi is the sample value of independent identical distribution, and the kernel function *K* is a weighting function. In this paper, the distribution pattern of eco-efficiency values of green buildings is estimated by the Gaussian kernel density function, and its function expression is shown in the above ② equation. To ensure the accuracy of kernel density estimation, a smaller *h* value is generally chosen, and the dynamic evolution information such as distribution and development trend of the observed object (eco-efficiency value) in time is examined by graphical comparison.

### 3.3. Moran's I Index Analysis

To study the spatial autocorrelation of green building eco-efficiency and explore the spatial correlation and clustering characteristics between the level of green building eco-efficiency in a certain region and its neighboring regions, this paper uses the global Moran's I index and local Moran's I index to test the green building eco-efficiency based on the spatial weight matrix of geographical distance. The global Moran's I index is usually used to measure the global spatial distribution characteristics of the object under examination, which can better reflect whether there is spatial clustering and other characteristics of the object under observation. The local Moran's I index, on the other hand, reflects whether there is spatial agglomeration characteristics and spatial correlation behavior of the object under examination with high or low observed values in different regions, and the calculation formula is as follows:

(5) $$\begin{array}{c} \text{global: }I=\frac{\sum_{i=1}^{n}\sum_{j=1}^{n}W_{ij}\left(x_{i}-\bar{x}\right)\left(x_{j}-\bar{x}\right)}{S^{2}\sum_{i=1}^{n}\sum_{j=1}^{n}W_{ij}},\\ \text{local: }I_{i}=\frac{\left(x_{i}-\bar{x}\right)}{S^{2}}\sum_{j=1}^{n}W_{ij}\left(x_{j}-\bar{x}\right), \end{array}$$

where *n* is the number of samples; *x*_*i*_ and *x*_*j*_ are the green building eco-efficiency values of province and city *i* and province and city *j*; *w*_*ij*_ is the spatial weight matrix, and this paper uses the geographic distance spatial weight matrix; $\bar{x}$, *s*^2^ are the mean and variance of green building eco-efficiency of each province and city, respectively; global situation *I* > 0 indicates a positive spatial correlation, *I* < 0 indicates a negative spatial correlation, and *I* = 0 indicates no spatial correlation.

## 4. Indicator Selection and Data Sources

### 4.1. Input-Output Index Selection

Drawing on the idea of sustainable development strategy elaborated by Damato et al. [52], green building eco-efficiency can be interpreted as the ratio of the output of building value (economic value, ecological value) to the input of resources. Therefore, based on the current situation of green building development in China, the index requirements of the data envelope model, and the availability of data, this paper selects capital, labor, energy, land, technology, and other factors as input indicators, and economic and environmental factors as output indicators, so as to construct the green building eco-efficiency evaluation index system (see Table 1). Among them, all the data can be obtained directly or indirectly from the statistical yearbook, except for the carbon emission data, which cannot be obtained directly, while the carbon emission calculation is mainly referred to the IPCC carbon emission accounting method and related research results [53, 54].

### 4.2. Selection of External Environmental Variables

Environmental variables are used in the SFA regression model of stage 2, and factors that have an impact on the eco-efficiency of green buildings but are not subjectively controlled by the construction industry are mainly selected [55]. Combining the current situation of China's construction industry development, the sustainable development driving characteristics of green buildings, and relevant research data, and after considering the limitations of the research model and objective factors, this paper focuses on the environmental variables that affect the eco-efficiency of green buildings from four levels: economic level, urban proportion, scientific and technological support, and energy structure (Table 2).

Level of economic development: the level of eco-efficiency of green buildings is limited by the level of regional economic development. Macroeconomic differences are a key factor causing regional differences in the development of the construction industry, which has an important impact on the management of construction production and technology supply. In this paper, regional GDP per capita is chosen to characterize the level of regional economic development.

Level of urbanization: the urbanization process drives the population to move to cities and towns, which to a certain extent affects the supply and demand of the construction industry and also has a certain environmental impact on urban construction. Therefore, this paper uses the proportion of urban population in the total population of a region to characterize the impact of the level of urbanization.

Science and technology support: the level of regional investment in science and technology is crucial to the development and application of green technologies. The adoption of advanced green technologies and management experience can optimize and improve the building production process, which is an important means to achieve energy saving and emission reduction in buildings and promote the development of green buildings. In this paper, the proportion of regional investment in science and technology to fiscal expenditure is used to characterize the level of regional support for science and technology.

Energy structure: the energy consumption structure directly affects the carbon emission efficiency of the construction industry, and a reasonable optimization of the energy structure can effectively improve the low-carbon and green development of the construction industry. China's energy structure is dominated by coal, and the proportion of coal consumption to total energy consumption is chosen in this paper to characterize the preference of building energy consumption.

### 4.3. Data Sources

In this paper, 30 Chinese provinces (regions and cities, excluding Tibet, Hong Kong, Macao, and Taiwan) are selected as the research objects, and the panel data of input-output and environmental variables from 2013 to 2020 are used to measure the eco-efficiency of green buildings in each province and city, and the studied regions are divided into eastern, central, and western based on geographical location and other factors to facilitate the analysis of their regional differences. The data were obtained from the China Statistical Yearbook, China Construction Statistical Yearbook, China Energy Statistical Yearbook, and the statistical yearbooks of each province and city in the relevant years. The descriptive statistical characteristics of the input-output sample data are shown in Table 3, which shows that the standard deviation and extreme deviation of individual indicators are large, indicating the existence of large differences, and the input and output situations also reflect large differences.

## 5. Empirical Research

### 5.1. Analysis of Green Building Eco-Efficiency Measurement Results

There are significant differences in green building eco-efficiency across Chinese provinces and municipalities, and the specific efficiency results only consider the influence of the green building industry's own development in different regions, while ignoring the actual external environmental variables and random errors that interfere with it. Therefore, it does not reflect the actual level of green building eco-efficiency in each province and city, so it is necessary to measure the efficiency by placing different provinces and cities under the same environmental conditions. Therefore, using the level of economic development, urbanization level, technological support, and energy structure as independent variables and the slack value of input variables as dependent variables, the SFA regression was measured using Frontier 4.1 software based on equation (2), and the data required were the arithmetic mean of the variables from 2013 to 2020, and the measured results are shown in Table 4.

As can be seen from Table 4, the likelihood ratio LR for each variable passed a mixed chi-square test with a significance level of 5% or 1% over the period 2013–2020, indicating that the external environmental variables selected for this paper would have a significant impact on the green building eco-efficiency measure and that it is reasonable to conduct an SFA regression analysis. And the values of each variable were close to 1 and passed the significance test, indicating that the management inefficiency factor accounts for a large proportion of the total variance, while the effect of random error is limited, indicating that the use of the SFA regression model is necessary. The regression coefficients of the four external environmental variables on the five input slack variables were able to pass the significance level tests of 10%, 5%, and 1%, indicating that the external environmental variables had different degrees of influence on the input slack variables.

The input slack variable is the difference between the actual input of each decision unit and the target (optimal efficiency state) input, that is, the amount of waste of the input of each decision unit. When the coefficient of the environmental variable is negative, it means that an increase in the external environmental variable will reduce the input slack variable; that is, it will help reduce the waste of the input slack variable and achieve an increase in relative efficiency; when the coefficient of the environmental variable is positive, it means that an increase in the external environmental variable will increase the input slack variable; that is, it will increase the waste of the input slack variable and cause a decrease in relative efficiency.

1. Level of economic development: the level of economic development is positively correlated with the slack variables of each input and reaches a significance level of 5%, 1%, 1%, 5%, and 10%, respectively. This indicates that an increase in the level of economy can reduce the redundancy of inputs of capital, labor, energy, land, and technology, which is conducive to the improvement of eco-efficiency of green buildings and is a dominant external environmental factor.
2. Level of urbanization: the level of urbanization is positively correlated with the rate of technological equipment and fixed asset investment and negatively correlated with the other three, with high significance. This indicates that the increase in the level of urbanization causes an increase in input redundancy in technology and capital, while at the same time suppressing input redundancy in labor, energy, and land. Clearly, urbanization is bound to cause certain economic, social, and environmental pressures, and the development of green buildings and their scaling up will effectively improve the eco-efficiency of the industry.
3. Science and technology support: the effect of scientific and technological support on labor force and housing construction land area is positive, while the effect on the remaining three items is negative, all reaching a significance level of 1%. This generally indicates that expenditure on science and technology can create a good green technological environment and has a positive effect on improving the eco-efficiency of green buildings, but attention needs to be paid to the effective allocation of resources while strengthening technological research and development.
4. Energy structure: the energy structure has efficiency advantages for energy consumption and fixed asset investment, which can suppress the input redundancy of energy and capital but is positively correlated with technology and equipment rate and labor, which can increase the input redundancy of technology and labor, while the redundancy of housing construction land area is not significant.

The above analysis shows that different external environment variables and random errors have different effects on the slack values of each input, which may cause different development environments and opportunities for the green building industry in each region and thus lead to the eco-efficiency of green building in each province and city being contrary to the actual situation. Therefore, based on the SFA regression results to adjust each original input, all decision units were placed under the same external environment and random error state to examine a more realistic level of efficiency.

Therefore, the provinces and cities were adjusted to the same external environment and random error, and the input variables were adjusted according to equation (3), and based on the superefficient SBM model, the MAXDEA software was used to analyze the efficiency of the adjusted input data and the original output data to measure the final green building eco-efficiency of each province and city in China. The results of the mean green building eco-efficiency measures for Stages 1 and 3 were obtained (Table 5). It can be seen that there are significant regional differences in the eco-efficiency of green buildings in the eastern, central, and western regions of China, with the eastern efficiency value in stage one (0.884) being greater than the national average (0.724), and 20.3% and 34.6% higher than those in the central (0.704) and western (0.578) regions, respectively, and expanding to 27.1% and 39.7% in stage three, which clearly shows that the central and western construction companies have a far more inefficient management of green buildings than in the east, but the positive effect of their external environment makes up for some of the regional disparity.

Although the change in the average value of efficiency for each region before and after the adjustment is relatively small, there is a large gap in green building eco-efficiency between provinces and municipalities at the interprovincial level. The number of regions on the frontier of green building eco-efficiency increased from six to seven, with Shandong, Guangdong, Henan, and Shaanxi changing from non-DEA effective to DEA effective, and Beijing, Hubei, and Chongqing changing from DEA effective to non-DEA effective, and the efficiency ranking of each province and city changed significantly before and after adjustment, possibly due to measurement errors in the data or the external environment such as the scale of regional green building construction and the high or low level of development. Therefore, SFA regression analysis was used in Stage 2 to remove the external environment and random errors in order to obtain relatively true efficiency values.

### 5.2. Analysis of Temporal Differences in Eco-Efficiency of Green Buildings

#### 5.2.1. Analysis of Temporal Differences in Green Building Eco-Efficiency

Based on the analysis of the three-stage superefficiency SBM model above, the final measurement results of green building eco-efficiency in each province and city from 2013 to 2020 were obtained (Table 6), and the changing trend and coefficient of variation of green building eco-efficiency in each region were plotted (Figure 1), according to which the temporal variation analysis of green building eco-efficiency in China was conducted.

1. From the overall change, China's green building eco-efficiency showed steady growth during 2013–2020, and after a brief increase and then decrease fluctuation during 2013–2016, its efficiency value continued to rise, with an overall average annual increase of 5.64%, but the national average value was only 0.701, indicating that the national green building industry and its eco-function were on the middle level, still 30% away from the efficiency frontier surface. There is still 30% room for improvement. And the coefficient of variation is characterized by a U-shaped evolution until 2015, falling from 0.587 in 2013 to 0.402 in 2016, and rising to 0.461 in the following year before sliding to 0.405 in 2020, with an average annual decrease of 5.17%. This is accompanied by the national strategy of green building and new urbanization background, and the regions pay attention to green building development and urban ecological construction, strengthen the ecological environment management in the construction field, and play a certain positive role in green building eco-efficiency, but due to the ecological drawbacks of large-scale construction and urban expansion emerge, the gap between the production input and eco-efficiency frontier surface of green building in China still needs to be improved urgently.
2. From the interprovincial level, only seven provinces, namely, Shanghai, Jiangsu, Zhejiang, Shandong, Guangdong, Henan, and Shaanxi, have reached the DEA effective mean value of green building eco-efficiency from 2013 to 2020, and the rest of the provinces and cities have not reached the frontier surface. The green building eco-efficiency values for both Jiangsu and Guangdong are greater than 1 for each year of the study period, indicating that their resource input and sustainable development of green buildings maintain good coordination and are national benchmark regions. Among the many non-DEA effective provinces and cities, Hubei (0.954) and Beijing (0.963) are in a dominant position and have a high level of green building development; Hebei, Sichuan, and Guizhou have annual average growth rates of more than 10%, which are higher than the highly efficient regions such as Beijing and Shanghai, showing a significant ecological catch-up effect; Heilongjiang, Inner Mongolia, Qinghai, Ningxia, and Xinjiang have long-term input. The effect is not obvious, and its efficiency change tends to be stable but ranked at the bottom, while the ecological efficiency of green buildings in Chongqing and Shaanxi continues to rise. Obviously, there are significant interprovincial differences in green building eco-efficiency.
3. In terms of regions, the efficiency of the east (0.895) is greater than the national average and far exceeds that of the central (0.653) and western (0.540) regions, showing a development pattern of “east > central > west,” and the overall trend of green building eco-efficiency in the three regions is similar, all showing growth. The overall trend of green building eco-efficiency in the east shows an M-shaped fluctuation, and the efficiency value increases from 0.787 in 2013 to 1.021 in 2020, with an average annual increase of 3.79%; the central green building eco-efficiency continues to rise from 2013 to 2016 to the first wave (0.672) and then shows a V-shaped fluctuation, with an average annual increase of 6.30%; the western green building eco-efficiency increases from 2013 to 2017 and then leveled off with an average annual increase of 8.59%. The coefficients of variation of green building eco-efficiency in the east, central, and west decreased by 39.47%, increased by 2.56%, and increased by 59.01% overall, respectively. Obviously, although the level of eco-efficiency of developing green buildings varies significantly among individual provinces and cities, the regional gap has slightly narrowed.

#### 5.2.2. Time Evolution Trend Analysis of Green Building Eco-Efficiency

To explore the temporal development of green building eco-efficiency in China and its dynamic characteristics, this paper uses stata15.0 to estimate the kernel density of green building eco-efficiency in China from 2013 to 2020 and selects 2013, 2015, 2017, and 2020 to draw kernel density curves (Figure 2) to compare and study its temporal evolution pattern.

1. In terms of distribution position, the center of the density function for four years shows a trend of moving to the right, indicating that the eco-efficiency of green buildings in China is gradually increasing, among which the rightward shift in 2013, 2015, and 2017 is not obvious enough, which indicates that the improvement of eco-efficiency of green buildings in China is limited during this period, while the rightward shift in 2020 is larger compared with the previous years, reflecting the fact that since then, China's green building eco-efficiency has increased rapidly after a slow growth. The reason for this is the promotion of national policies such as new urbanization, energy saving, and emission reduction in buildings and the 13th Five-Year Plan for Green Buildings in the past few years, which has led to an explosion in the scale of green buildings and the promotion of urban ecological civilization.
2. In terms of distribution patterns, China's green building eco-efficiency experienced an evolutionary process from bimodal distribution to single peak and from sharp peak to broad peak during 2013–2020, with a steeper wave in 2013 and a bimodal structure, and a more concentrated and significant polarization of green building eco-efficiency during this period, mainly manifesting as a decrease in the degree of concentration while the national green building eco-efficiency increased the “catch-up effect” of low-efficiency provinces and cities (Yunnan, Gansu, etc.) on high-efficiency provinces and cities (Hebei, Tianjin, etc.), which is insufficient; the years 2015–2020 all show a single-peak distribution and a continuous decline in the peak, and the span of the interval gradually increases, indicating that the overall regional gap expands and shows obvious dynamic dispersion characteristics.
3. In terms of peak changes, the peak of the density function from 2013 to 2020 shows a significant decline, and the corresponding nuclear density value of the left peak in 2013 is significantly larger than that of the right peak, which indicates that the peak areas in that year are mostly concentrated in low-efficiency areas; that is, the number of low-efficiency areas is much higher than that of high-efficiency areas; the peak from 2015 to 2020 gradually decreases, and the center of the density function shifts significantly to the right, and its corresponding efficiency value increases significantly. This indicates that the overall eco-efficiency of green buildings in China has increased significantly, but the number of provinces and cities with increased efficiency has decreased.

### 5.3. Analysis of Spatial Differences in Eco-Efficiency of Green Buildings

#### 5.3.1. Spatial Distribution Pattern of Green Building Eco-Efficiency

To fully characterize the evolution of the spatial pattern of green building eco-efficiency in China, ArcGIS10.6 was used to visualize the green building eco-efficiency of each province and city from 2013 to 2020, and the efficiency was divided into low-efficiency zones (0, 0.4), medium-low efficiency zones [0.4, 0.6], medium-efficiency zones [0.6, 0.8], medium-high efficiency zones [0.8, 1.0], and high-efficiency zones (1.0 and above) in five gradations, and intercepted 2013, 2015, 2017, and 2020 as time sections to obtain the spatial distribution map of eco-efficiency of green buildings in China (Figure 3).

In general, the spatial pattern of green building eco-efficiency in China from 2013 to 2020 shows an obvious “transitional” distribution pattern, showing a gradient diffusion from the eastern region to the western region. The eco-efficiency of green buildings in most provinces and cities has increased to different degrees during the study period, and the polarization difference is significant, and the overall pattern shows a gradual transition from the medium-low efficiency zone to the medium-medium efficiency zone. Among them, in 2013, the ecological efficiency of green buildings in China was generally below the medium-low development level and showed a polarization pattern dominated by the medium-low scale, with low-efficiency zones (all western regions except Shaanxi and Chongqing and some central and eastern regions) account for about 46.7% of the country; medium-low and lower efficiency zones account for a total of 76.7%, concentrated in the west and most of the central region, while the medium-high efficiency zone was only scattered in seven provinces and cities in the middle and east; in 2015, most of the central and southwest regions Green building eco-efficiency showed a small increase, and the east and central regions gradually showed a multitype mixture, with more than medium-efficiency areas concentrated in the east and Henan and Hubei provinces, and medium-low and below-efficiency areas distributed in northern and southwestern provinces and cities; in 2017, the number of green building eco-efficiency low-efficiency areas decreased significantly, and medium-high and above-efficiency areas increased significantly, which obviously promoted the regional green building greatly in that year as a national strategy the growth of eco-efficiency, among which Shaanxi, Chongqing, Shandong, and Shanghai were transformed from medium, medium, medium-high, and medium-efficient zones to high-efficiency zones, and medium-efficient zones were gradually concentrated in the central region. In 2020, the ecological efficiency of green buildings showed a nonequilibrium characteristic of transition with the high-efficiency zone in Shandong, Jiangsu, Zhejiang, and other eastern coastal areas as the core, gradually decreasing to the central (medium-middle-high mixed efficiency zone) and western zones (northwest, northeast, and due north low-efficiency zone).

#### 5.3.2. Spatial Clustering Characteristics of Green Building Eco-Efficiency

From the previous analysis, it can be seen that there may be some dependency on the characteristics of green building eco-efficiency differences among regions. To further explore the spatial aggregation effect and diffusion characteristics of regional green building eco-efficiency, this paper measures Moran's I index of green building eco-efficiency and its correlation test values from 2013–2020 with the help of GeoDa software (Table 7), and the results show that Moran's I index of green building eco-efficiency in China during the study period is positive, shows small growth fluctuations, and passes the 5% (*P* < 0.05, *Z* > 1.96). This indicates that the spatial pattern of interprovincial green building eco-efficiency is not randomly distributed, but there is a continuous positive spatial correlation and agglomeration feature, and this feature is steadily increasing over time, which is similar to the pattern of regional economic development in China in recent years.

Based on the local Moran scatter plots of green building eco-efficiency in Chinese provinces and cities drawn in 2013 and 2020 (Figure 4), the spatial agglomeration state of green building eco-efficiency in each province and city and its evolution characteristics are further revealed.

Among the agglomeration types, the provincial and municipal ratios of high-high type (H-H), low-high type (L-H), low-low type (L-L), and high-low type (H-L) are 8 : 9:10 : 3 and 10 : 7:11 : 2 in 2013 and 2020, respectively, and it is obvious that the areas in H-H and L-L types are the most, accounting for 60% and 70%, an increase of 16.7%, indicating that the spatial homogeneity of green building eco-efficiency is gradually increasing, while the spatial heterogeneity is gradually decreasing; that is, high-efficiency regions tend to be adjacent to high-efficiency regions and low-efficiency regions tend to be adjacent to low-efficiency regions, and the difference in polarized distribution continues to expand. Types of local agglomeration distribution by region corresponding to scatter diagram can be seen in Table 8.

1. H-H type agglomeration area (the first quadrant) mainly includes Shanghai, Shandong, Jiangsu, Zhejiang, and other eastern coastal areas and some central China (Henan, Hubei) and northwest China (Shaanxi), indicating that these areas pay attention to the coordinated development of urban construction and new urbanization, have a high level of green building development and advanced urban ecological concepts, and drive each other, so that the improvement of their own efficiency has a positive radiation and diffusion effect on the neighboring areas. Tianjin leaps from L-H type to H-H type, and it is obvious that it has a significant advantage of “being diffused” and is influenced and driven by the neighboring provinces and cities with high ecological efficiency of green building during the study period. The spatial difference with neighboring high-efficiency regions has been reduced, and the region has been ranked among the high-efficiency regions.
2. The L-H agglomeration area (the second quadrant) mainly covers some provinces and cities in the southwest, northwest, and central regions, where the development level of green buildings and new urbanization is low; the L-L agglomeration area (the third quadrant) mainly includes the less developed regions in the central and western regions and the northeast region, which have more room for improvement, but the growth rate is slow. Among them, although Jiangxi and Anhui are adjacent to the high-efficiency region, they cannot be driven to the H–H agglomeration. On the contrary, Hainan, Anhui, and Hunan are negatively radiated by their near neighbors and show a relative displacement from L-H to L-L type. Sichuan and Heilongjiang leap from L-L to L-H, playing the advantage of “driven” location and steadily improving their green building eco-efficiency. In contrast, Inner Mongolia, Liaoning, Jilin, Guangxi, and other regions maintain the same L-L agglomeration state in 2013 and 2020, because these regions are relatively lagging in their own green building technology and its development, and the scale of the industry is insufficient and lacks regional competitiveness, which leads to an imbalance in their green building eco-efficiency inputs and outputs and makes it difficult to break away from the inefficient agglomeration development mode, and these regions should pay attention to improving the green building management level and input resource allocation ability.
3. H-L type agglomeration area (fourth quadrant) includes Hebei, Chongqing, and Guangdong in 2013 and Hebei and Chongqing in 2020. Guangdong, as a developed region along the southeast coast, ranks among the top in the country in terms of green building eco-efficiency, but its regional cogovernance mechanism of the construction industry chain is poor and did not produce effective positive radiation to neighboring regions in 2013, while the polarization phenomenon of high local green building eco-efficiency and low neighboring regions emerged. However, Guangdong itself has strong green science and technology innovation capital and achieved a leap from H-L to H–H in 2020 after actively promoting the concept of green building and low-carbon development of the construction industry. The green building eco-efficiency of Chongqing and Hebei has grown steadily, but the economic status of their provincial construction industry and its special green building capacity is lagging behind the national average and is vulnerable to the influence of the surrounding environment, leaping to the junction of H-L and L-L and the junction of H-L and H-H, respectively.

## 6. Conclusion

This paper measures the green building eco-efficiency of Chinese provinces and cities from 2013–2020 based on the three-stage superefficiency SBM-DEA model, reveals the differences and evolutionary characteristics of green building eco-efficiency in the temporal and spatial dimensions, and obtains the following conclusions.

1. China's green building eco-efficiency showed a stable growth during 2013–2020, with an average annual increase of 5.64% and an average annual decrease of 5.17% in the coefficient of variation, but the national average value was only 0.701, indicating that the national green building industry and its eco-function were on the middle level, and the overall efficiency differences over the years narrowed over time; the overall pattern showed “East > Central > West” development pattern, and although the difference in efficiency level between individual provinces and cities is significant, the regional gap is slightly reduced, which is accompanied by the national strategy of green building and new urbanization background, and each region attaches importance to green building development and urban ecological construction and strengthens ecological environment management in the construction field, which plays a certain positive role in green building ecological efficiency, but because the ecological drawbacks of large-scale construction and urban expansion have emerged, the gap between China's green building production input and the ecological efficiency frontier still needs to be improved urgently.
2. The kernel density function curve of green building eco-efficiency reflects the process of slow growth and then rapid improvement of green building eco-efficiency in China during the study period and undergoes the evolution process from double-peak distribution to single-peak and from sharp peak to broad peak, showing that the concentration of high-efficiency regions decreases, while green building eco-efficiency increases, the number of provinces and cities with efficiency growth decreases, and the overall absolute difference of regional efficiency is narrowed and shows obvious dynamic dispersion characteristics; the “transitional” spatial distribution pattern of green building eco-efficiency is remarkable, and the overall gradient development trend is gradually transitioned from medium-middle low-efficiency area to medium-middle high-efficiency area. For this reason, China should implement the local governance of green building, give full play to the local comparative advantages, coordinate and improve the supporting policies of green building and its related industries, and promote the common development of regional green building eco-efficiency by increasing the degree of internal and external development between provinces, enhancing the technical exchanges between provinces and cities, and clarifying the regional development direction.
3. The results of spatial autocorrelation show that there is a continuous positive spatial correlation and agglomeration characteristic of green building eco-efficiency, and this characteristic is steadily enhanced over time; the spatial spillover and diffusion effect of high-efficiency regions is significant, and the low-efficiency regions generally maintain a low growth trend, showing an improvement in the bipolar distribution characteristics, but the interprovincial gap is still huge; the green building eco-efficiency of most regions has “Matthew effect,” showing significant spatial agglomeration and path dependence and generally presenting the spatial club convergence characteristics that developed regions tend to be H-H agglomeration type and less developed regions tend to be L-L aggregation type. For this reason, China should devote itself to breaking the geographical limitation of ecological efficiency development of green buildings, forming a situation where the upstream high-efficiency level areas are driven by radiation and the middle and downstream low-efficiency level areas are developed in a linkage; local governments should deepen interregional technical cooperation and division of labor, enhance the ability of the central and western low-efficiency provinces and cities to absorb the spillover effects of the eastern high-efficiency provinces and cities, and form a green sharing situation of open competition and win-win cooperation, so as to narrow the geographical gap and improve the ecological efficiency level of green buildings in China.

## Figures and Tables

**Figure 1:** Trends and coefficient of variation of eco-efficiency of green buildings by region, 2013–2020. (a) Efficiency mean. (b) Coefficient of variation.

**Figure 2:** Kernel density distribution of eco-efficiency of green buildings.

**Figure 3:** Spatial distribution of eco-efficiency of green buildings in China.

**Figure 4:** Green building eco-efficiency local Moran scatter plot (2013, 2020).

**Table 1:** Green building eco-efficiency evaluation indexes.

Indicator categories		Indicator name	Indicator meaning
Input indicators	Capital input	Fixed asset investment in construction industry (billion)	Reflecting the capital investment in the construction industry
	Labor input	Number of employees in construction industry enterprises (person)	Reflecting the manpower qualified to participate in green building projects
	Energy input	Total energy consumption (million/ t standard coal)	Reflecting the green production capacity of the construction industry
	Land input	Building area of houses (million m^2^)	Reflecting the construction of land for green building projects
	Technical input	Technical equipment rate (yuan/person)	Reflecting the level of green technology and equipment application of green building

Output indicators	Expected output	Total construction industry output value (billion yuan) Total profit of construction industry enterprises (million yuan)	Reflecting the economic output of green building
	Unexpected output	Carbon emissions (million tons)	Reflecting the environmental output of green building

**Table 2:** External environmental variables for eco-efficiency in green buildings.

	Variable name	Variable values	Variable description
Environment variables	Economic level	GDP per capita (billion yuan)	Measuring the impact of the level of regional economic development
	Urban share	Urban population share of total population (%)	Measuring the impact of regional urbanization level
	Technology support	Regional investment in science share of fiscal expenditure (%)	Measuring the impact of green technology support and R&D
	Energy structure	Coal consumption share of total energy consumption (%)	Measuring building energy consumption preferences

**Table 3:** Results of descriptive statistics of input-output variables of the sample (2013–2020).

Variable	Sample	Max.	Min.	Average	Standard deviation
Fixed asset investment in construction industry (billion)	240	1136.86	0.09	131.45	201.44
Number of employees in construction industry enterprises (person)	240	8110275	54847	1604115.18	1785021
Total energy consumption (million/t standard coal)	240	354.33	14.91	126.23	75.88
Building area of houses (million m^2^)	240	249176.80	738.96	39362.64	47499.82
Technical equipment rate (yuan/person)	240	91231.43	728	14354.99	9978.62
Total construction industry output value (billion yuan)	240	6717.06	52.22	1211.13	1302.94
Total profit of construction industry enterprises (million yuan)	240	11617738	64449	2093927.95	2070219
Carbon emissions (million tons)	240	52901.55	562	13178.71	11055.73

**Table 4:** SFA regression results.

Independent variable	Technical equipment rate slack variables	Workforce slack variables	Fixed asset investment slack variables	Building site area slack variables	Energy consumption slack variables
Constant term	−1.34*E* + 04^*∗∗∗*^	2.14*E* + 06^*∗∗∗*^	−1.27*E* + 02^*∗∗∗*^	4.28*E* + 04^*∗∗∗*^	4.89*E* + 01^*∗∗∗*^
	(−2.30*E* + 03)	(3.13*E* + 04)	(−1.27*E* + 02)	(9.65*E* + 03)	(4.89*E* + 01)

Economic level	−5.02*E* − 02^*∗∗*^	−2.52*E* + 01^*∗∗∗*^	−4.72*E* + 01^*∗∗∗*^	−5.97*E* + 01^*∗∗*^	−1.81*E* − 03^*∗*^
	(−2.86*E* + 00)	(4.72*E* + 00)	(−7.04*E* + 00)	(2.46*E* + 00)	(1.88*E* + 00)

Urban share	2.39*E* + 02^*∗∗*^	−7.74*E* + 04^*∗∗∗*^	6.86*E* + 00^*∗∗∗*^	−2.01*E* + 03^*∗∗∗*^	−2.74*E* + 00^*∗∗∗*^
	(2.02*E* + 00)	(−3.24*E* + 01)	(1.23*E* + 01)	(−1.29*E* + 01)	(−2.74*E* + 00)

Technology support	−1.18*E* + 03^*∗∗∗*^	4.43*E* + 05^*∗∗∗*^	−1.42*E* + 01^*∗∗∗*^	1.39*E* + 04^*∗∗∗*^	−4.16*E* + 00^*∗∗∗*^
	(−1.05*E* + 02)	(3.59*E* + 03)	(−1.42*E* + 01)	(1.84*E* + 03)	(−4.16*E* + 00)

Energy structure	9.49*E* + 01^*∗∗*^	6.62*E* + 03^*∗*^	−2.35*E* + 00^*∗∗∗*^	−2.81*E* + 01	−2.86*E* + 01^*∗∗*^
	(2.10*E* + 00)	(−1.75*E* + 00)	(−2.86*E* + 00)	(−1.42*E* − 01)	(2.21*E* + 00)

*σ* ^2^	7.58*E* + 07^*∗∗∗*^	1.00*E* + 12^*∗∗∗*^	2.83*E* + 04^*∗∗∗*^	9.51*E* + 08^*∗∗∗*^	2.99*E* + 03^*∗∗∗*^
	(7.58*E* + 07)	(1.00*E* + 12)	(2.83*E* + 04)	(9.51*E* + 08)	(2.99*E* + 03)

*γ*	1.00*E* + 00^*∗∗∗*^	9.60*E* − 01^*∗∗∗*^	1.00*E* + 00^*∗∗∗*^	1.00*E* + 00^*∗∗∗*^	1.00*E* + 00^*∗∗∗*^
	(1.08*E* + 04)	(2.52*E* + 01)	(1.06*E* + 05)	(1.50*E* + 05)	(2.05*E* + 01)

Log	−2.96*E* + 02	−4.39*E* + 02	−1.72*E* + 02	−3.33*E* + 02	−1.44*E* + 02

LR	1.11*E* + 01^*∗∗*^	8.90*E* + 00^*∗∗*^	2.14*E* + 01^*∗∗∗*^	1.22*E* + 01^*∗∗*^	1.14*E* + 01^*∗∗*^

*Note*. ^*∗∗∗*^, ^*∗∗*^, ^*∗*^ represent tests passing significance levels of 1%, 5%, and 10% respectively; the test values for *T* are in brackets.

**Table 5:** Mean measurement results of eco-efficiency of green buildings in stages 1 and 3.

Region		Phase 1		Phase 3	
		Efficiency value	Sort	Efficiency value	Sort
East	Beijing	1.267	4	0.963	8
	Tianjin	0.636	17	0.643	12
	Heibei	0.436	24	0.797	11
	Liaoning	0.882	8	0.539	20
	Shanghai	1.330	3	1.062	4
	Jiangsu	1.543	1	1.371	1
	Zhejiang	1.409	2	1.137	3
	Fujian	0.468	22	0.620	14
	Shandong	0.550	19	1.027	6
	Guangdong	0.667	12	1.196	2
	Hainan	0.534	20	0.492	24
	Average	**0.884**	—	**0.895**	—

Middle	Shanxi	0.650	14	0.559	18
	Jilin	0.572	18	0.564	17
	Heilongjiang	0.654	13	0.372	27
	Anhui	0.413	26	0.545	19
	Jiangxi	0.873	9	0.594	15
	Henan	0.923	7	1.046	5
	Hubei	1.045	6	0.954	9
	Hunan	0.504	21	0.589	16
	Average	**0.704**	—	**0.653**	—

West	Neimenggu	0.772	11	0.365	28
	Guangxi	0.421	25	0.525	21
	Chongqing	1.206	5	0.841	10
	Sichuan	0.814	10	0.639	13
	Guizhou	0.641	15	0.523	22
	Yunnan	0.445	23	0.513	23
	Shanxi	0.637	16	1.002	7
	Gansu	0.288	30	0.461	25
	Qinghai	0.347	29	0.327	30
	Ningxia	0.411	27	0.352	29
	Xinjiang	0.379	28	0.392	26
	Average	**0.578**	—	**0.540**	—

National average		**0.724**	—	**0.701**	—

**Table 6:** Final measurement results of eco-efficiency of green buildings in each city and province.

Region	2013	2014	2015	2016	2017	2018	2019	2020	Average
Beijing	0.973	1.021	0.839	0.923	0.856	1.076	0.944	1.068	0.963
Tianjin	0.379	0.522	0.532	0.576	0.584	0.757	0.874	0.919	0.643
Heibei	0.384	0.591	0.678	0.691	0.928	1.014	1.086	1.006	0.797
Liaoning	0.450	1.037	0.461	0.580	0.521	0.510	0.316	0.436	0.539
Shanghai	0.927	1.113	0.946	1.028	1.066	1.125	1.111	1.183	1.062
Jiangsu	1.572	1.131	1.336	1.000	1.601	1.419	1.341	1.566	1.371
Zhejiang	1.227	1.117	0.999	1.148	1.311	1.101	1.030	1.163	1.137
Fujian	0.420	0.572	0.660	0.484	0.614	0.662	0.734	0.812	0.620
Shandong	0.882	0.840	0.969	1.097	1.077	1.002	1.142	1.207	1.027
Guangdong	1.078	1.284	1.138	0.980	1.222	1.346	1.221	1.299	1.196
Hainan	0.362	0.381	0.453	0.488	0.558	0.537	0.585	0.569	0.492
East	**0.787**	**0.874**	**0.819**	**0.818**	**0.940**	**0.959**	**0.944**	**1.021**	**0.895**
Shanxi	0.338	0.358	0.574	0.601	0.427	0.638	0.701	0.835	0.559
Jilin	0.461	0.588	0.554	0.449	0.585	0.642	0.675	0.558	0.564
Heilong jiang	0.358	0.240	0.388	0.383	0.366	0.434	0.422	0.381	0.372
Anhui	0.428	0.535	0.471	0.457	0.613	0.576	0.581	0.699	0.545
Jiangxi	0.469	0.514	0.586	0.706	0.441	0.573	0.711	0.750	0.594
Henan	0.855	1.008	1.032	1.155	0.970	1.080	1.036	1.234	1.046
Hubei	0.525	0.902	0.878	1.043	0.929	1.140	1.270	0.948	0.954
Hunan	0.558	0.578	0.519	0.580	0.582	0.492	0.684	0.716	0.589
Middle	**0.499**	**0.590**	**0.625**	**0.672**	**0.614**	**0.697**	**0.760**	**0.765**	**0.653**
Neimenggu	0.352	0.318	0.362	0.409	0.360	0.377	0.354	0.390	0.365
Guangxi	0.363	0.416	0.543	0.635	0.522	0.565	0.567	0.588	0.525
Chongqing	0.470	0.557	0.689	0.883	1.010	1.081	1.077	0.961	0.841
Sichuan	0.342	0.654	0.540	0.635	0.724	0.655	0.772	0.792	0.639
Guizhou	0.231	0.400	0.478	0.588	0.573	0.575	0.554	0.783	0.523
Yunnan	0.352	0.482	0.521	0.496	0.599	0.544	0.568	0.543	0.513
Shanxi	0.572	0.769	0.791	0.962	1.284	1.186	1.237	1.214	1.002
Gansu	0.399	0.403	0.328	0.405	0.581	0.473	0.534	0.566	0.461
Qinghai	0.281	0.357	0.242	0.230	0.305	0.491	0.374	0.338	0.327
Ningxia	0.288	0.380	0.353	0.373	0.322	0.341	0.388	0.375	0.352
Xinjiang	0.270	0.382	0.336	0.414	0.391	0.481	0.438	0.427	0.392
West	**0.356**	**0.465**	**0.471**	**0.548**	**0.606**	**0.615**	**0.624**	**0.634**	**0.540**
National	**0.552**	**0.648**	**0.640**	**0.680**	**0.731**	**0.763**	**0.778**	**0.811**	**0.701**

**Table 7:** Green building eco-efficiency global Moran's I index, 2013–2020.

Year	2013	2014	2015	2016	2017	2018	2019	2020
Moran's I	0.213	0.226	0.219	0.236	0.227	0.244	0.253	0.271
*P*-value	0.001	0.023	0.008	0.017	0.011	0.024	0.036	0.021
Z-value	2.471	2.235	3.211	3.640	2.095	2.706	2.537	3.314

**Table 8:** Types of local agglomeration distribution by region (2013, 2020).

Year	2013	2020
H-H type	Shanghai, Shandong, Jiangsu, Zhejiang, Henan, Hubei, Shaanxi, Beijing	Shanghai, Shandong, Jiangsu, Zhejiang, Henan, Hubei, Shaanxi, Beijing, Guangdong, Tianjin
L-H type	Guizhou, Yunnan, Gansu, Jiangxi, Xinjiang, Tianjin, Hainan, Anhui, Hunan	Guizhou, Yunnan, Gansu, Jiangxi, Xinjiang, Sichuan, Heilongjiang
L-L type	Neimenggu, Liaoning, Jilin, Guangxi, Shanxi, Fujian, Ningxia, Qinghai, Sichuan, Heilongjiang	Neimenggu, Liaoning, Jilin, Guangxi, Shanxi, Fujian, Ningxia, Qinghai, Sichuan, Heilongjiang
H-L type	Hebei, Chongqing, Guangdong	Hebei, Chongqing, Guangdong

## Data Availability

The data used to support the findings of this study are available from the corresponding author upon request.
